The article "Highly Expressed lncRNA GAS5 in the Serum of Children with Mycoplasma pneumoniae Pneumonia and Its Effect on LAMPs-Induced Apoptosis and Inflammation" was published in 2022. Journal: Contrast Media Mol Imaging.

# Highly Expressed lncRNA GAS5 in the Serum of Children with *Mycoplasma pneumoniae* Pneumonia and Its Effect on LAMPs-Induced Apoptosis and Inflammation

**DOI:** 10.1155/2022/7872107

**Published:** 2022-08-09

**Authors:** Juhua Ji, Lei Song, Fei Hong, Weiyan Zhang, Meijun Zhu, Xiaohong Yang, Chuangli Hao

**Affiliations:** ^1^Children's Hospital of Soochow University, No. 92 Zhongnan Street, Wuzhong District, Suzhou, Jiangsu 215000, China; ^2^Department of Pediatrics, The Second Affiliated Hospital of Nantong University, Nantong First People's Hospital, No. 6, North Haierxiang Road, Nantong 226001, China

## Abstract

The aim of the study was to explore the serum expression of long noncoding RNA (lncRNA) growth arrest-specific transcript 5 (GAS5) in *Mycoplasma pneumoniae* pneumonia (MPP) and its effect on lipid-associated membrane proteins (LAMPs)-induced apoptosis and inflammation. Totally, 56 children with MPP (MPP group) and 56 healthy children (NC group) were enrolled. lncRNA GAS5 expression was measured by quantitative real-time polymerase chain reaction (qRT-PCR). Serum levels of tumor necrosis factor *α* (TNF-*α*) and interleukin-6 (IL-6) were detected using ELISA, and the high mobility family protein B1 (HMGBl) was detected by qRT-PCR. The methylated binding protein 2 (MECP2) was inhibited by gene silencing, and the expression of MECP2, TNF-*α*, IL-6, HMGBl, p-p65, and p-I*κ*B*α* was measured. lncRNA GAS5 and TNF-*α*, IL-6, and HMGBl in the peripheral blood of the MPP group were positively correlated (*P* < 0.05). The expression of TNF-*α*, IL-6, HMGBl, and lncRNA GAS5 showed a positive correlation with that of LAMPs. The GAS5-siRNA group showed an increased cell survival rate compared with the scrambled-RNAi group (*P* < 0.05) while showing decreased apoptosis and cell death rates (*P* < 0.05). In addition, the expression of IL-6, TNF-*α*, HMGBl, p-p65, and p-I*κ*B*α* was significantly reduced (*P* < 0.05). lncRNA GAS5 is highly expressed in the serum of children with MPP and inhibits LAMPs-induced apoptosis and alveolar macrophage inflammation.

## 1. Introduction

*Mycoplasma pneumoniae* pneumonia (MPP) is one of the common types of community-acquired pneumonia in children. Although it is self-limiting and most cases can be cured with a good prognosis, some cases are further aggravated, developing into severe pneumonia, and endangering the lives of children [1]. A study has shown [2] that humoral immunity, cellular immunity, and cytokines contribute to the development of MPP. Long noncoding RNAs (lncRNAs) are a group of regulatory RNAs consisting of 200 nucleotides that mediate a variety of cellular physiological processes such as chromatin structure, transcriptional and posttranscriptional processes, and intracellular transport [3]. Growth arrest-specific transcript 5 (GAS5) is a lncRNA that encodes a small nucleolar RNA host gene [4]. Some transcripts of lncRNA GAS5 bind to the glucocorticoid receptor (GR) and prevent its activation, thereby preventing hormonal regulation of its target genes. lncRNA GAS5 is crucial to the diagnosis and treatment of bronchial asthma [5]. Glucocorticoid is an important clinical treatment for refractory MPP (RMPP). It has been found that GR*α* is predominantly expressed in MPP and RMPP, especially in RMPP [6]. Therefore, we speculated that GAS5 might play a role in the treatment of MPP by combining with GR. However, the role of lncRNA GAS5 in MPP has not yet been explored. Lipid-associated membrane proteins (LAMPs) are structural lipid-related membrane proteins present in mycoplasma and play an important role in the interaction between mycoplasma and the host. Recent studies have shown that LAMPs stimulate human monocytes and macrophages in vitro, which can induce the expression of proinflammatory cytokines such as interleukin-1*β* (IL-1*β*) and interleukin-6 (IL-6) and activate the nuclear factor-kappa B (NF-*κ*B) to induce apoptosis of cells [7]. The apoptotic effect of LAMPs on host cells directly affects the occurrence and development of MPP, which is an important component of mycoplasma pathogenicity. In this study, LAMPs were used to stimulate mouse alveolar macrophage cell line MH-S to inhibit the lncRNA GAS5 expression through siRNA silencing to observe its effect on the expression of inflammatory factors secreted by MH-S, providing basic information on inflammatory lung diseases.

## 2. Materials and Methods

### 2.1. General Data

Totally, 56 children with MPP were assigned to the MPP group, including 34 males and 22 females, aged 1–12 years, with a mean age of (4.69 ± 1.22) years. Inclusion criteria were as follows: (1) children who met the MPP diagnostic criteria in practical pediatrics; (2) children who were not receiving relevant treatment before admission; (3) children who were free of other pathogenic infections such as viruses and bacteria; (4) children who were free of immune system diseases; and (5) those whose consent form was signed by family members. Exclusion criteria were as follows: (1) patients with congenital diseases such as congenital heart disease and congenital malformations; (2) patients with malignant tumors; (3) patients with hepatic and renal insufficiency; (4) patients with a combination of psychiatric disorders; and (5) patients with a combination of severe endocrine diseases. Meanwhile, 56 healthy children were selected for the normal control (NC) group, including 36 males and 20 females, aged 1–12 years, with a mean age of (4.49 ± 1.13) years. This study was approved by the medical ethics committee of Children's Hospital of Soochow University.

### 2.2. Methods

#### 2.2.1. Expression of lncRNA GAS5, TNF-*α*, IL-6, and HMGBl in Peripheral Blood

Peripheral blood samples were collected from MPP and NC groups and centrifuged at 3000 r/min for 20 min, and the serum was collected. The levels of IL-6 and TNF-*α* were detected using enzyme-linked immunosorbent assay (ELISA) kits (Hangzhou Unitech Biotechnology Co., Ltd., Hangzhou, China) and a Model 550 microplate reader (Bio-Rad, Hercules, CA, USA) was used to detect the OD values of the corresponding factors. The total RNA from the serum was extracted, cDNA was obtained by reverse transcription, PCR was performed with GAPDH as the internal reference, and the lncRNA GAS5 and HMGB1 levels were measured using quantitative real-time polymerase chain reaction (qRT-PCR).

#### 2.2.2. MH-S Cell Culture and Transfection

Mouse alveolar macrophage MH-S cells (Cell Bank of Chinese Academy of Sciences, Shanghai, China) were cultured in Dulbecco's modified eagle medium-high glucose (Gibco, Rockville, MD, USA) with 10% fetal bovine serum (Sigma-Aldrich, St. Louis, MO, USA) under the following conditions: 37°C, 5% CO_2_ saturated humidity. Cell passaging was performed when the cells were in the logarithmic phase of growth and at approximately 80–90% confluence. The second-passage cells were taken for subsequent experiments. MH-S cells were used to prepare a single cell suspension and inoculated with a density of 1.0–2.0 × 10^5^/ml to the plate. After incubation for 24 h, the plate was washed three times with PBS. The cells were divided into four groups: in the control group, cells were cultured under normal conditions without any intervention; in the LAMPs group, cells were treated with LAMPs (Invitrogen, Carlsbad, CA, USA) to establish a cell injury model; in the scrambled-RNAi group, si-NC was transfected into MH-S cells and stimulated with LAMPs; and in the GAS5-siRNA group, si-GAS5 was transfected into MH-S cells and stimulated with LAMPs. lncRNA GAS5 interfering fragment and overexpression vector were purchased from Shanghai Gemma Pharmaceutical Technology Co., Ltd. (Shanghai, China).

#### 2.2.3. Detection of the lncRNA GAS5 Expression

Total RNA was extracted from treated MH-S cells using Trizol reagent (Invitrogen, Carlsbad, CA, USA), cDNA was obtained by reverse transcription using a Reverse Transcription System Reverse Transcription Kit (Promega, Madison, WI, USA), and the expression was determined through a qRT-PCR instrument (Thermo Fisher Scientific, Waltham, MA, USA) with GAPDH as the internal reference. GAPDH primer sequence: upstream 5′-CACCCTCAAGATCATCAGCA-3′, downstream 5′-TGTGGTCATGAGTCCTTCCA-3′, amplification length: 106 bp. GAS5 primer sequence: upstream 5′-CTTGCCTGGACCAGCTTAAT-3′, downstream 5′-CAAGCCGACTCTCCATACCT-3′, amplification length: 122 bp. All PCR primers were purchased from Shanghai Shengong Bioengineering Co., Ltd. (Shanghai, China). The reaction system was 25 *μ*l. SYBR Green was mixed. The reaction conditions were as follows: 95°C predenaturation for 15 s, 95°C denaturation for 10 s, 60°C annealing for 20 s, and 72°C extensions for 15 s over 40 cycles. The gene expression was calculated using the 2-∆∆ct method.

#### 2.2.4. Detection of Apoptosis

MH-S cells were transfected for 72 h and washed with PBS. Cells were resuspended and the cell density was adjusted to 2 × 10^5^/ml. Then, 195 *μ*L of the cell suspension was added into the detection tube, treated with 5 *μ*L of Annexin V-FITC (BioVision, Milpitas, CA, USA), incubated for 15 min, washed, and centrifuged at 1000 r/min for 3 min. Cells were resuspended, treated with propidium iodide (BioShop, Canada), and incubated for 15 min, followed by detecting the apoptosis using flow cytometry.

#### 2.2.5. Detection of the Protein Expression of TNF-*α* and IL-6

The supernatant of the treated MH-S cells was centrifuged at 3000 r/min for 20 min, and the protein expression of TNF-*α* and IL-6 was detected by ELISA according to the kit instructions.

#### 2.2.6. Detection of the Expression of p-p65 and p-I*κ*B*α*

Treated MH-S cells were mixed with 400 *μ*l of RIPA (PMSF, 100 mmol/L) (Shanghai Zeye Biotechnology Co., Ltd., Shanghai, China) and placed on ice for 30 min, followed by centrifugation at 4°C, 12000 r/min for 30 min. The supernatant was treated with SDS-PAGE protein loading buffer and denatured at 100°C for 10 min. SDS-PAGE gel electrophoresis (Bio-Rad electrophoresis instrument, Borel, Hercules, CA, USA) was performed and the membrane was incubated in 5% skimmed milk and sealed at room temperature for 3 h. The membrane was washed with TBST. Primary antibodies (p-p65, p-I*κ*B*α*, and I*κ*B*α* antibodies, Cell Signaling, Danvers, MA, USA) were added and incubated at 4°C overnight, followed by washing with TBST three times and adding a secondary antibody (horseradish peroxidase-tagged secondary antibody, Beijing Solarbio Science & Technology Co., Ltd., Beijing, China) for incubation at 37°C for 1 h. The expression of p-p65 and p-I*κ*B*α* was analyzed by ImageJ software using *β*-actin as the internal reference.

#### 2.2.7. Statistical Analysis

Data processing was performed using Statistical Package for Social Science (SPSS) 25.0 software (IBM, Armonk, NY, USA) and measurement data were expressed as *x̅* ± *s*, with a one-way ANOVA for comparison among three groups and LSD *t*-test for comparisons between two groups. The test level was *α* = 0.05 and all tests were two-sided. The Pearson correlation was used to analyze the correlation between lncRNA GAS5 and TNF-*α*, IL-6, and HMGBl. *P* < 0.05 indicates a significant difference.

## 3. Results

### 3.1. Comparison of Baseline Data

There was no significant difference in sex and age between the two groups (*P* > 0.05), indicating comparability (Table 1).

### 3.2. Expression of lncRNA GAS5, TNF-*α*, IL-6, and HMGBl in Peripheral Blood

The expression levels of lncRNA GAS5, TNF-*α*, IL-6, and HMGBl in the peripheral blood of the MPP group were significantly higher than those in the NC group (*P* < 0.05). Correlation analysis showed that the lncRNA GAS5 expression showed a significant positive correlation with the expression of TNF-*α*, IL-6, and HMGBl in the MPP group (rTNF-*α* = 0.482, PTNF-*α* < 0.001; rIL-6 = 0.571, PIL-6 < 0.001; rHMGBl = 0.466, PHMGBl < 0.001). This suggests that lncRNA GAS5, TNF-*α*, IL-6, and HMGBl are expressed at higher levels in MPP patients, and the level of lncRNA GAS5 was significantly positively correlated with the level of inflammatory cytokines (Figure 1).

### 3.3. Expression of TNF-*α*, IL-6, HMGB1, and lncRNA GAS5 after Stimulation of LAMPs in MH-S Cells

MH-S cells were treated with 0, 125, 250, 500, 1000, and 2000 ng/mL of LAMPs; then, the gene expression was assessed by q-PCR. The expression of TNF-*α*, IL-6, HMGBl, and lncRNA GAS5 were all significantly increased and gradually increased with the increasing LAMPs concentration (*P* < 0.05). In subsequent experiments, 1000 ng/mL of LAMPs were used as the final concentration to stimulate MH-S cells (Figure 2).

### 3.4. Role of lncRNA GAS5 in MH-S Cells and Its Effect on the Survival Rate of LAMPs-Induced MH-S Cells

To investigate the role of lncRNA GAS5 in MH-S cells, lncRNA GAS5-siRNA was used to silence the lncRNA GAS5 expression. In the GAS5-siRNA group, the lncRNA GAS5 expression was significantly lower compared to that of the scrambled-RNAi group (*P* < 0.05), suggesting lncRNA GAS5 was successfully inhibited in MH-S cells (Figure 3(a)). The MTT method was used to detect the survival rate of LAMPs-induced MH-S cells. The LAMPs and scrambled-RNAi groups showed a decreased cell survival rate compared with that of the control group (*P* < 0.05). Besides, the GAS5-siRNA group showed an increased cell survival rate compared with that of the scrambled-RNAi group (*P* < 0.05, Figure 3(b)). These results suggest that downregulation of lncRNA GAS5 can inhibit LAMPs-induced macrophage necrosis.

### 3.5. Effect of lncRNA GAS5-siRNA on LAMPs-Induced Apoptosis in MH-S Cells

LAMPs and scrambled-RNAi groups had a higher apoptosis rate compared to that of the control group (*P* < 0.05); the apoptosis rate of MH-S cells in the GAS5-siRNA group was significantly lower (*P* < 0.05) compared to that of the scrambled-RNAi group, suggesting that downregulation of the lncRNA GAS5 expression inhibits LAMPs-mediated induction of MH-S cell apoptosis (Figure 4).

### 3.6. Effect of lncRNA GAS5-siRNA on the LAMPs-Induced Inflammatory Response in MH-S Cells

Compared to the scrambled-RNAi group, the GAS5-siRNA group expressed IL-6, TNF-*α*, and HMGBl at low levels (*P* < 0.05), suggesting that inhibition of lncRNA GAS5 can reduce LAMPs-induced secretion of inflammatory cytokines (Figure 5).

### 3.7. Effect of lncRNA GAS5-siRNA on the LAMPs-Induced Protein Expression of p-p65 and p-I*κ*B*α* in MH-S Cells

Compared to the LAMPs group, the protein levels of p-p65 and p-I*κ*B*α* in the GAS5-siRNA group were decreased (*P* < 0.05), suggesting that lncRNA GAS5 may inhibit LAMPs-induced secretion of inflammatory cytokines by downregulating the expression of NF-*κ*B pathway-related proteins (Figure 6).

## 4. Discussion

MPP accounts for 10–40% of all childhood pneumonia [8, 9], and it induces the humoral immune response and promotes the synthesis and release of immunoglobulins as well as the formation of immune complexes. Surface antigens of MPP could alter the levels of some cell surface antigens, inducing immune cells, causing them to attack host tissues and cause immune dysfunction [10, 11]. lncRNAs play a crucial role in immune responses [12]. GAS5 is a single-stranded noncoding RNA that is mainly located in the cytoplasm, though it can be transported to the nucleus under certain conditions, and GAS5 can inhibit GR activation and regulate the target genes expression through miRNAs [13–18].

TNF-*α* and IL-6 are highly expressed in inflammatory lung diseases [19, 20]. HMGBl is predominantly distributed in eukaryotic cells and mediates late inflammatory responses through its release into the extracellular compartment [21, 22]. Overexpression of GAS5 exacerbates the secretion of oxidized low-density lipoprotein (ox-LDL)-induced proinflammatory cytokines IL-6, IL-1*β*, and TNF-*α* in macrophages [23].

The present study showed increased levels of lncRNA GAS5, TNF-*α*, IL-6, and HMGBl in the peripheral blood of children with MPP. Further, the expression level of lncRNA GAS5 was correlated with that of TNF-*α*, IL-6, and HMGB1, suggesting that the lncRNA GAS5 expression is closely related to that of inflammatory cytokines and HMGBl, consistent with the results of above studies. Our further experiments showed that after stimulation with varying concentrations of LAMPs, the mRNA and protein expression levels of lncRNA GAS5, TNF-*α*, IL-6, and HMGB1 all gradually increased dose-dependently (*P* < 0.05). These results indicate that lncRNA GAS5 may be related to the secretion of inflammatory factors in MH-S cells.

Exogenous lncRNA GAS5 can regulate apoptosis in macrophages and endothelial cells in atherosclerosis [24]. lncRNA GAS5 may serve as a target for controlling cell apoptosis through the control of inflammation. Our results showed that after inhibiting the expression of lncRNA GAS5 by siRNA silencing, the expression level of lncRNA GAS5 in MH-S cells was decreased, the survival rate of MH-S cells was significantly increased, and the expression levels of IL-6, TNF-*α*, and HMGBl were decreased significantly, indicating that inhibition of the expression of lncRNA GAS5 could regulate the apoptosis of MH-S cells, decrease the release of inflammatory factors, and inhibit the HMGB1 level.

The NF-*κ*B pathway is an important signal transduction system in inflammatory lung diseases and can be involved in the body's inflammatory response, immune response, and apoptosis upon activation [25, 26]. In the resting state, NF-*κ*B and I*κ*B form inactive complexes present in the cytoplasm. After cells are stimulated by bacterial lipopolysaccharide and cytokines, I*κ*B exposes p65, the nuclear localization site of NF-*κ*B, causing its phosphorylation. This activates the NF-*κ*B pathway, promotes the release of inflammatory factors, and mediates the involvement of various cytokines in the process of lung injury [27]. Results revealed that the protein expression of p-p65 and p-I*κ*B*α* was significantly reduced in cells with silenced lncRNA GAS5 (*P* < 0.05), showing that lncRNA GAS5 may regulate the release of inflammatory factors and HMGBl in MH-S cells by inhibiting the activation of the NF-*κ*B pathway. It has been indicated that the NF-*κ*B P65 expression level was increased in mice with MPP and was involved in immune damage caused by mycoplasma infection [28], consistent with the results of this study.

However, there are still some deficiencies in this study. The small number of cases in this study and the fact that it was a single-center study may have caused some bias in the results. In the next study, the number of cases will be increased, and a multicenter study will be conducted to validate the findings of this study. In addition, the downstream mechanism of the effect of lncRNA GAS5 on MMP has not been further investigated in this study and will be actively explored in the next study.

## 5. Conclusions

In summary, lncRNA GAS5 is highly expressed in the serum of children with MPP and inhibits LAMPs-induced apoptosis and inflammation in alveolar macrophages, possibly through the inhibition of NF-*κ*B activation. However, the specific mechanism underlying this phenomenon needs to be further investigated.

## Figures and Tables

**Figure 1:** Comparison of lncRNA GAS5 and cytokine expression in children with MPP (mean ± SD, *n* = 56). (a) TNF-*α*; (b) IL-6; (c) HMGB1; and (d) lncRNA GAS5. Compared with the NC group, ^*∗∗∗*^*P* < 0.001. lncRNA GAS5: long noncoding RNA growth arrest-specific transcript 5; MPP: *Mycoplasma pneumoniae* pneumonia; TNF-*α*: tumor necrosis factor *α*; IL-6: interleukin-6; HMGB1: mobility family protein B1.

**Figure 2:** Changes in the expression of inflammatory factors after LAMPs stimulation in MH-S cells (mean ± SD, the experiment was repeated three times). (a) TNF-*α*; (b) IL-6; (c) HMGBl; and (d) lncRNA GAS5. Compared with the NC group at the same time point, ^#^*P* < 0.05, ^###^*P* < 0.001. LAMPs: lipid-associated membrane proteins; TNF-*α*: tumor necrosis factor *α*; IL-6: interleukin-6; HMGB1: mobility family protein B1; lncRNA GAS5: long noncoding RNA growth arrest-specific transcript 5.

**Figure 3:** Validation of the lncRNA GAS5 interference expression vector and its effect on the survival rate of LAMPs-induced MH-S cells (mean ± SD, the experiment was repeated three times). (a) Validation of the lncRNA GAS5 interference expression vector; (b) effect of lncRNA GAS5-siRNA inhibition on the survival rate of LAMPs-induced MH-S cells. Compared with the NC group, ^*∗∗∗*^*P* < 0.001; compared with the LAMPs group, ^###^*P* < 0.001; compared with the scrambled-RNAi group, ^&&&^*P* < 0.001. lncRNA GAS5: long noncoding RNA growth arrest-specific transcript 5; LAMPs: lipid-associated membrane proteins.

**Figure 4:** Effect of lncRNA GAS5-siRNA on LAMPs-induced apoptosis in MH-S cells (mean ± SD, the experiment was repeated three times). (a) Flow cytograms of MH-S cell apoptosis and (b) bar graphs showing the comparison of apoptosis rates. Compared with the control group, ^*∗∗∗*^*P* < 0.001; compared with the LAMPs group, ^###^*P* < 0.001; compared with the scrambled-RNAi group, ^&&&^*P* < 0.001. lncRNA GAS5: long noncoding RNA growth arrest-specific transcript 5; LAMPs: lipid-associated membrane proteins.

**Figure 5:** lncRNA GAS5-siRNA inhibits LAMPs-induced inflammatory responses in MH-S cells (mean ± SD, the experiment was repeated three times). (a) TNF-*α*; (b) IL-6; and (c) HMGBl. Compared with the control group, ^*∗∗∗*^*P* < 0.001; compared with the LAMPs group, ^###^*P* < 0.001; compared with the scrambled-RNAi group, ^&&&^*P* < 0.001. lncRNA GAS5: long noncoding RNA growth arrest-specific transcript 5; LAMPs: lipid-associated membrane proteins; TNF-*α*: tumor necrosis factor *α*; IL-6: interleukin-6; HMGB1: mobility family protein B1.

**Figure 6:** lncRNA GAS5-siRNA inhibits LAMPs-induced protein expression of p-p65 and p-I*κ*B*α* in MH-S cells (mean ± SD, the experiment was repeated three times). (a) Western blots of p-p65 and p-I*κ*B*α* protein expression in MH-S cells; (b) bar graphs of p-p65 and p-I*κ*B*α* protein expression. (1) Control group; (2) LAMPs group; (3) scrambled-RNAi group. Compared with the control group, ^*∗∗∗*^*P* < 0.001; compared with the LAMPs group, ^###^*P* < 0.001. lncRNA GAS5: long noncoding RNA growth arrest-specific transcript 5; LAMPs: lipid-associated membrane proteins.

**Table 1:** Comparison of baseline data between the two groups (mean ± SD)/(*n*).

Group	Sex (male/female)	Mean age (years)
MPP group	34/22	4.69 ± 1.22
NC group	36/20	4.49 ± 1.13
*χ*2/*t*	0.152	0.900
*P*	0.696	0.370

## Data Availability

The datasets used and analyzed during the current study are available from the corresponding author upon reasonable request.
